The article "The clinical features of 590 patients with brucellosis in Xinjiang, China with the emphasis on the treatment of complications" was published in 2017. Journal: PLoS Negl Trop Dis.

# The clinical features of 590 patients with brucellosis in Xinjiang, China with the emphasis on the treatment of complications

**DOI:** 10.1371/journal.pntd.0005577

**Published:** 2017-05-01

**Authors:** Bin Jia, Fengbo Zhang, Ying Lu, Wenbao Zhang, Jun Li, Yuexin Zhang, Jianbing Ding

**Affiliations:** 1 Department of Infection Disease Center, The First Affiliated Hospital of Xinjiang Medical University, Urumqi, Xinjiang, China; 2 Department of Clinical Laboratory, The First Affiliated Hospital of Xinjiang Medical University, Urumqi, Xinjiang, China; 3 Department of Respiratory and Respiratory Intensive Care Unit Center, The First Affiliated Hospital of Xinjiang Medical University, Urumqi, Xinjiang, China; 4 Department of Immunology, Basic Medical College, Xinjiang Medical University, Urumqi, China; King Saud University College of Medicine, SAUDI ARABIA

## Abstract

**Background:**

This study aims to analyze the clinical characteristics and treatment outcomes of 590 patients with brucellosis in Xinjiang, China.

**Methodology and principal findings:**

The clinical characteristics, laboratory findings, complications and prognosis of 590 patients infected with brucellosis were retrospectively analyzed. These patients had a mean age of 44.24 ± 15.83 years with 60.5% having a history of close contacting with cattle and sheep. Of them, 53.6% (316 /590) were in acute phase and 21.5% were in chronic phase. Agglutination test showed 98.5% positive with 34% blood culture positive of *Brucella*. The major symptoms were fatigue (91%), hyperhidrosis(88.1%), fever(86.9%), and joint pain(81%) with 29.8% having enlarged liver, 26.1% having enlarged spleen and 23.2% having osteoarticular complications. Combination of doxycycline plus rifampicin for 12 weeks was an effective regimen for patients without complications. The 3-drug regimen (doxycycline+rifampicin+levofloxacin) for 12 weeks was recommended for these with complications. There were 6 patients died (1.02%) with overall relapse rate of 5.98%.

**Conclusions:**

Brucellosis is mostly associated with contacting with domestic animal production in Xinjiang, China. Clinical symptoms include fever, fatigue, hyperhidrosis, and joint pain with common complication of osteoarticular involvement. Three-drug-regimen of doxycycline+rifampicin+levofloxacin for 12 weeks was effective for these patients with complications.

## Author summary

Brucellosis is a highly contagious zoonosis caused by bacteria of the genus Brucella and affecting mammals. Human Brucellosis is caused by ingestion of unpasteurized or undercooked food product from infected animals, or close contact with them. The infection with same bacteria even with same type can lead to manifestations varying from patient to patient. And there is no consensus for treating all types of brucellosis. In this paper, we retrospectively reviewed symptoms of Brucellosis in 590 patients living in Xinjiang area of China. We found that the percentage of chronic Brucellosis in Xinjiang from our study was 23.5%, which was higher than previous report. The reason for this increasing can be further explored. We also suggest that, despite the WHO recommended first-line 2-drug regimen is effective and preferred in most cases, the 3-drug regimen of doxycycline+rifampin+levofloxacin for 12 weeks should be recommended for patients with complications or experienced prolonged treatment. These findings are of clinical significance to improve Brucellosis management.

The article "The clinical features of 590 patients with brucellosis in Xinjiang, China with the emphasis on the treatment of complications" was published in 2017. Journal: PLoS Negl Trop Dis.

## Introduction

Brucellosis (or undulant fever) is a zoonotic disease with a worldwide distribution, mainly in the Mediterranean Basin, Middle East, Central and South America, and Asia [1]. Xinjiang Uygur Autonomous Region (Xinjiang) in western China is an agricultural area with animal production as its major primary industry. The incidence of brucellosis is high in this region [2] with prevalence being 9.80/100000, 17.51/100000, and 33.02/100000 in 2012, 2013, and 2014, respectively [3]. The disease is transmitted to humans through closely contacting with sick animals or consumption of raw meat and dairy products [4]. Patients may present with fever, sweating, fatigue, and osteoarticular pain [5]. The major systemic complications of the disease involve osteoarticular involvement[6], cardiological and neurological disorders. The incidence of endocarditis disease is about 2%, however, it accounts for 80% of brucellosis related death [5]. The combination of antibiotics is the main regimen for brucellosis [7]. Long-term of taking drugs is required for cure treatment and reducing relapsed cases [8].

In this study, the clinical features of 590 cases with brucellosis and their treatment were retrospectively analyzed.

## Materials and methods

### Ethics statement

A written informed consent was obtained from every patient and the study was approved by the Ethics Committee of The First Affiliated Hospital of Xinjiang Medical University.

### Patients

Patients diagnosed with brucellosis from 2005 to 2015 in The First Affiliated Hospital of Xinjiang Medical University were recruited. The diagnosis of brucellosis was based on medical history, clinical features, positive serum agglutination tests and/or blood cultures [9]. The patient’s presentation was categorized as acute phase (with symptoms less than 3 months), subacute phase (3–6 months) and chronic phase (more than 6 months). The blood was cultured using automatic blood culture system (France Biomerieux Co. Ltd., Bact / ALERT 3D 60) with an average incubation time of 5–7 days according to the method described by Tabibnejad [10]. The pathogen of positive culture was identified using automatic microbial identification machine (France Biomerieux Co. Ltd., VITEK 2 COMPACT 30). The clinical presentations, laboratory results and treatment outcome were recorded.

The article "The clinical features of 590 patients with brucellosis in Xinjiang, China with the emphasis on the treatment of complications" was published in 2017. Journal: PLoS Negl Trop Dis.

### Signs and symptoms

The initial signs and symptoms of brucellosis cases include fever, sweats, malaise, anorexia, headache, pain in muscles, joint, and/or back and fatigue. The complications of brucellosis cases include osteoarticular, endocarditis, epididymalorchitis, nervous disorders, and liver involvement. The diagnosis of endocarditis was based on the revised diagnostic criteria of DUKE infective endocarditis [11], presenting as valve vegetation on transthoracic echocardiography or transesophageal echocardiography. The epididymalorchitis was diagnosed by epididymal testicular pain and positive ultrasound findings. Liver involvement or liver damage refers to increased alanine aminotransferase and aspartate aminotransferase (more than 2 times of the normal upper limit) of laboratory tests, excluding other reasons. The diagnosis of nervous disorder included culture of Brucella using cerebrospinal fluid as gold standard and/or neurological symptoms and abnormal cerebrospinal fluid examination.

### Laboratory tests

Blood was collected from patients for testing ALT, AST, GGT, ALP, TBil and Alb measured by biochemical analyzer (Roche cobas8000). A complete blood count was determined on the Sysmex XN2000 analyzer. The erythrocyte sedimentation rate (ESR) was detected using Wechsler method. The C-reactive protein (CRP) was detected using the immune turbidimetric method (Beckman immage800). The standard tube agglutination antigen was purchased from the Institute of Infectious Diseases, China Center for Disease Control and Prevention. Blood culture was performed for these patients with symptom of chilling or their body temperature over 38.5°C before use of antimicrobial drugs.

### Treatment

Chemotherapeutical regimens combined with two or three drugs were employed for treating these patients with different presentations and conditions. These combinations were doxycycline+rifampicin, doxycycline+levofloxacin, doxycycline+streptomycin and doxycycline+rifampicin+levofloxacin. The doses for orally taking these drugs were doxycycline, 100 mg p.o., every 12 hours; rifampin,600 mg p.o., once per day; streptomycin, 1 g intramuscular injection, once per day, and levofloxacin, 500 mg p.o, once per day. For some reasons, we also prescribed the second-line drugs for some patients included levofloxacin (500 mg p.o, once per day), cotrimoxazole (960 mg p.o,twice per day), ciprofloxacin (750 mg p.o, twice per day) and ceftriaxone (2g ivgtt, once per day). All patients were treated for 12 weeks and followed up for 6 months. Positive clinical symptoms and physical examinations indicated disease recurrence.

The article "The clinical features of 590 patients with brucellosis in Xinjiang, China with the emphasis on the treatment of complications" was published in 2017. Journal: PLoS Negl Trop Dis.

### Statistical analysis

The data were analyzed using SPSS software (Version 17.0, SPSS Inc., Chicago, Ill., USA). The measurement data were expressed as mean ± standard deviation. T test and chi-square test were used to analyze the differences. P < 0.05 was statistically significant.

## Results

### Patient’s characteristics

A total of 590 patients were included in this study. Detailed demographics are shown in Table 1. Of them, 455 (77.1%) were male and 135 (22.9%) were female with mean age of 44.24 ±15.83 (3–75) years. There were 316 cases in acute phase, 136 cases in subacute phase, 127 cases in chronic phase and 11 showed no symptom but showing serological positive in agglutination test. Most(357, 60.5%)of the patients were farmers for raising cattle and sheep; and 145 (24.6%) cases had consumption history of dried raw meat or dairy products. There were 180 patients (30.5%) having different complications. All the patients were given 12 weeks of treatment. And since 2010, we gave those patients having complications three drugs combination regimen, doxycycline+rifampicin+levofloxacin, which significantly reduced relapsed cases compared to doxycycline+refampicin combination.

**Table 1:** Baseline demographics of patients with brucellosis.

Number of patients	590
Male	455 (77.1%)
Female	135 (22.9%)
Age (Average, years)	44.24 ±15.83
3–18 years	59 (10%)
19–45 years	292 (49.5%)
46–60 years	169 (28.6%)
61–75 years	70 (11.9%)
Staging	
Acute	316 (53.6%)
Subacute	136 (23.1%)
Chronic	127 (21.5%)
Asymptomatic	11 (1.86%)
Ethnicity	
Han	271 (45.9%)
Uighur	189 (32%)
Kazak	98 (16.6%)
Xibe	16 (2.71%)
Mongolia	9 (1.53%)
Hui	7 (1.19%)
Medical history	
Exposure and farming of cattle or sheep	357 (60.5%)
Consumption history of raw meat or dairy	145 (24.6%)
None	88 (14.9%)
History of complications	
Yes	180 (30.5%)
No	410 (69.5%)

### Clinical characteristics and complications

Table 2 shows the clinical characteristics of these patients including symptoms and complications were analyzed. These symptoms for the most patients were fever (86.9%), sweating (88.1%), fatigue (91%), and joint pain (81%). Some patients had back pain (54.6%), and shivers (52.5%). The most common signs of physical examinations were enlarged liver (176 cases, 29.8%), and enlarged spleen (154 cases, 26.1%). There were 137 cases (23.2%) with osteoarticular involvement, including 56 cases (40.9%) of sacroiliac arthritis, 48 cases (35%) of knee involvement, and 37 cases (27%) of spondylitis. There were 21 cases that involved the joints of ankle, elbow and shoulder, and, most of them were single joint involvement. There were 15 cases of epididymalorchitis,which is the most frequently involved of urinary and reproductive system.There were 10 cases (1.69%) complicated with endocarditis, including 8 cases (80%) of aortic valvular neoplasm.Fatigue,sweating and fever are the most common symptoms and osteoarticular system is most commonly involved.

The article "The clinical features of 590 patients with brucellosis in Xinjiang, China with the emphasis on the treatment of complications" was published in 2017. Journal: PLoS Negl Trop Dis.

**Table 2:** Clinical characteristics of patients with brucellosis.

Symptoms	Number of patients	%
Fatigue	537	91
Hyperhidrosis	520	88.1
Fever	513	86.9
Joint pain	478	81
Back pain	322	54.6
Anorexia	270	45.8
Weight loss	179	30.3
Nausea	78	13.2
Headache	46	7.80
Stomachache	21	3.56
Physical examinations		
Fever	300	50.8
Enlarged liver	176	29.8
Enlarged spleen	154	26.1
Scrotal swelling	15	2.54
Jaundice	3	0.51
Osteoarticular involvement	137	23.2
Genitourinary system involvement	15	2.54
Cardiovascular involvement	10	1.69
Pneumonia	6	1.02
Skin involvement	4	0.68
Nervous system involvement	1	0.17

### Laboratory tests

Table 3 shows the results of laboratory tests. There were 267 patients (45.3%) with anemia, 146 (24.7%) with abnormal white blood cells, 117(19.8%) with thrombocytopenia, 382 (64.7%) with elevated erythrocyte sedimentation rate (ESR) and 261 (44.2%) with increased C-reactive protein (CRP). The agglutination test antibody was positive (≥ 1:100) in 583 cases (99.8%) with highest antibody titer of 1: 1600. There were 179 patients (30.3%) with elevated transaminase. Totally 468 cases were tested by blood culture and 159 cases were positive (34%) of *Brucella melitensis*. The above suggest that elevated ESR and CRP are important laboratory indicators and that the blood culture needs to be improved.

**Table 3:** Laboratory results of patients with brucellosis.

	Number of patients	%
Anemia (Hb: male <14 mg / dl, Female < 12 mg / dl)	267	45.3
Lymphocytosis (lymphocytes > 45%)	197	33.4
Increased Transaminase (alanine/aspartame > 50 U / L)	179	30.3
Thrombocytopenia (platelets <15 × 10^4^ / mm^3^)	117	19.8
Leukocytosis (white blood cells > 10,000 / mm^3^)	91	15.4
Leukopenia (white blood cells < 4,000 / mm^3^)	55	9.3
Elevated ESR > (20 mm/h)	382	64.7
Increased CRP(> 8 mg/l)	261	44.2
Others		
Positive amber red plate test	590	100
Positive standard tube agglutination test (≥ 1: 100)	583	98.8
Positive culture (positive / all cases)	173/505	34.3
Blood culture	159/468	34.0
Bone marrow	12/31	38.7
Cardiac valve	2/3	66.7
Synovial fluid	0/2	0
Cerebral fluids	0/1	0

Note: Hb, hemoglobin; ESR, erythrocyte sedimentation rate; CRP, C-reactive protein.

The article "The clinical features of 590 patients with brucellosis in Xinjiang, China with the emphasis on the treatment of complications" was published in 2017. Journal: PLoS Negl Trop Dis.

### Treatment and prognosis

Table 4 shows the treatment and prognosis of these patients. Among the 590 patients, total of 468 patients were followed up. Fever is the symptom for the most patients, with 86.9% of the patients. When they received chemotherapeutical treatment, their body temperature returned to normal in 2–14 days after treatment with 85.2%(436/512) of the patients back to normal body temperature in one week. There were no significant differences in antipyretic effect among different treatment groups. For these patients without complications, relapse occurred in 10 patients (3.47%). There were 108 patients received without relapse in 6 months of follow-up.There was only one relapse (0.88%),less than the relapse rate of patients who received doxycycline+rifampin regimen for 6 weeks(3.30%).The patients took doxycycline+streptomycin and doxycycline+levofloxacin regimen, had higher relapse rate than doxycycline + rifampin regimen (P<0.05).

**Table 4:** Treatment plan, follow-up and prognosis.

	Number of cases (%)	Treatment duration (weeks)	Number of relapses (%)	Number of death
All patients in follow-up	468		28 (5.98)	6
Treatment plan (patients without complications)	288 (61.5)		10 (3.47)	1
Doxycycline + rifampicin	148	6–12	3 (2.03)	-
Doxycycline + levofloxacin	69	6–12	3 (4.35)	-
Doxycycline + streptomycin	51	6–12	2 (3.92)^b^	-
Doxycycline + ciprofloxacin	9	6–12	1 (11.1)	1
Doxycycline + ceftriaxone	11	6–12	1 (9.10)	-
Treatment plan (patients with complications)	180 (38.5)		17 (9.44)	-
Bone and joint complications	137		14 (10.2)^a^	-
Doxycycline + rifampicin	55	8–12	4 (7.27)	-
Doxycycline + streptomycin	11	8–12	2 (18.2%)^c^	1
Doxycycline + rifampin + levofloxacin	39	8–12	2 (5.13%)	-
Doxycycline + moxifloxacin	17	8–12	3 (17.6%)^c^	-
Rifampin + levofloxacin	15	8–12	3 (20)^c^	-
Endocarditis Complications	10 (2.14)			4
Doxycycline + rifampicin	1	8–12	2	2
Doxycycline + rifampicin + valve replacement	1	8–12	0	-
Doxycycline + rifampicin + ceftriaxone	2	8–12	1	1
Doxycycline + rifampin + ceftriaxone + valve replacement	3	8–12	0	-
Doxycycline + rifampin + levofloxacin	1	8–12	1	1
Doxycycline + rifampicin + levofloxacin + valve replacement	2	8–12	0	-

Note

a. There were significant differences of relapse rate between group with/ without osteoarticular complications (p < 0.05)

b. There were significant differences of relapse rate in doxycycline + streptomycin group between those with/ without osteoarticular complications (p < 0.05)

c. The relapse rate was higher in patients with osteoarticular complications receiving 2-drug regimen, compared with those receiving 3-drug regimen (p < 0.05).

The article "The clinical features of 590 patients with brucellosis in Xinjiang, China with the emphasis on the treatment of complications" was published in 2017. Journal: PLoS Negl Trop Dis.

For these patients with osteoarticular involvement, relapse was observed in 12 patients (8.76%), which is significantly higher than those without complications (3.47%) (p<0.05,Table 4). In addition, doxycycline+rifampicin regimen had the lowest relapse rate in patients without complications(p< 0.05). For those with osteoarticular complications, doxycycline+rifampicin+levofloxacin can have better treatment efficacy. All 10 cases with brucellosis endocarditis received had 3-drug regimen for 12 weeks. Among them, 6 cases had valve replacement surgery with good prognosis. The other 4 patients who did not received valve replacement surgery died from various reasons. These results indicate that doxycycline+rifampicin is a commonly used regimen with good efficacy for patients without complications. Combined use of doxycycline+rifampicin with levofloxacin is suitable for brucellosis patients with complications. We recommended 12 weeks continuous drug treatment.

## Discussion

Brucellosis has been increasingly becoming population health problem worldwide [12] in recent years. The number of brucellosis patients was increased yearly in our hospital in the last 10 years. During the hospital treatment, we found more patients had complications and at chronic stage. In the study, 23.5% of the 590 patients were at chronic phase, which is higher than other reports [4,13], indicating that more patients in Xinjiang were diagnosed improperly, which causes delayed treatment. Epidemiologically, contacting with animals and/or consumption of uncooked, disinfected milk and dairy products are the main risk factors for individuals having the infection [14]. Studies showed that 62.6–94.6% of patients in Turkey [15,16] and 79.1% of patients in Iran [17] ate raw or uncooked animal products. We showed that 24.6% of our patients were infected through consumption of raw and uncooked animal products, which is lower than those patients from other countries. From our clinical data, it showed that 66.9% of the patients came to our hospital in the months from March to May, which is also matched the published studies in Xinjiang, China[18,19]. In the pasture areas of Xinjiang, it is so called Spring lambing season from March to early May. In the season, sheep farmers take time to look after the new lambs The close contacting with ewes and new born lambs may be the main cause for the peak season of patients. In this study, there are 60.5% of patients closely contacted with cattle and sheep and 66.9% of the patients came to our hospital during the lambing season, indicating that helping lambing is the major activity or risk for infection.

The article "The clinical features of 590 patients with brucellosis in Xinjiang, China with the emphasis on the treatment of complications" was published in 2017. Journal: PLoS Negl Trop Dis.

In the study, 86.9% of brucellosis patients had fever. However, we found only 34% of those patients were blood culture positive, indicating blood bacteria may be not the main cause for fever. In addition, we found that the fever in all the patients was removed very quick once the patients took the drugs of doxycycline plus rifampicin. The fever was disappeared 2 or 14 days after taking antibiotics with the most (85.2%) back to normal in one week. It may be important for the doctors to make prescription in remote endemic areas, where diagnostic facility is poor. Doctor may give doxycycline+rifampicin to these patients with fever before identification of pathogen. in the endemic areas for diagnostic treatment. If the fever is down, it may indicate that the infection is brucellosis Antimicrobial therapy is the most effective treatment of brucellosis if patients are given right diagnosis.

The present study showed that the regimen of doxycycline+rifampin is suitable for these brucellosis cases without complications as recommended [17,20]. Patients given the doxycycline + levofloxacin regimen showed more relapse cases than doxycycline+rifampin regimen. However, we found that 3-drug regimen of doxycycline + rifampin + levofloxacin for osteoarticular complications showed very low relapse.

There are no consensus for treating neurobrucellosis including the regimen and course. The first-line regimen is doxycycline and rifampicin with or without aminoglycosides has been suggested[21–23]. We had one patient with meningitis who was successfully treated by doxycycline + rifampicin combined with ceftriaxone regimen for 6 months.

For these with brucellosis endocarditis, surgical treatment to replace valve should be performed for these patients with severe endocarditis if necessary. Maryam et al [24] showed that the mortality rate of brucellosis endocarditis with drug combined surgical treatment was 6.7% whereas that with drug treatment only was 32.7%. In our study, 10 patients with brucellosis endocarditis presented as fever, chest tightness, shortness of breath. Six patients were treated with antibiotics and valve replacement surgery with good prognosis. However, the other 4 patients without surgery died within 1-year of follow-up, indicating that the treatment of brucellosis endocarditis should include antibiotics and valve replacement surgery.

For patients at acute phase without complications, first-line drugs including doxycycline + rifampicin was recommended for 12 weeks. For patients with chronic course or complications, in addition to the first-line drugs, quinolones /cephalosporins should be added for at least for 12 weeks, thus completely removing pathogens in vivo, improving the cure rate and reducing relapse rate.

The article "The clinical features of 590 patients with brucellosis in Xinjiang, China with the emphasis on the treatment of complications" was published in 2017. Journal: PLoS Negl Trop Dis.

The serum agglutination test is a routing method for detecting antibodies in patients with brucellosis. Brucella bacteria culture is the "gold standard" for the diagnosis of brucellosis [25,26].

In conclusion, the epidemiological and medical history and clinical characteristics are crucial information in early and the differential diagnosis of brucellosis. WHO recommended first-line 2-drug regimen is still preferred; however, 3-drug regimen of doxycycline+rifampin+levofloxacin for 12 weeks is recommented for the patients with complications and at chronic stage.
